RETRACTED

# Biomechanical Characteristics of Hand Coordination in Grasping Activities of Daily Living

**DOI:** 10.1371/journal.pone.0146193

**Published:** 2016-01-05

**Authors:** Ming-Jin Liu, Cai-Hua Xiong, Le Xiong, Xiao-Lin Huang

**Affiliations:** 1 Institute of Rehabilitation and Medical Robotics, State Key Lab of Digital Manufacturing Equipment and Technology, Huazhong University of Science and Technology, Wuhan, Hubei 430074, China; 2 Foisie School of Business, Worcester Polytechnic Institute, Worcester, MA 01609–2280, United States of America; 3 Tongji Hospital, Tongji Medical College of Huazhong University of Science and Technology, Wuhan, Hubei 430030, China; Ohio State University Medical Center, UNITED STATES

## Abstract

Hand coordination can allow humans to have dexterous control with many degrees of freedom to perform various tasks in daily living. An important contributing factor to this important ability is the complex biomechanical architecture of the human hand. However, drawing a clear functional link between biomechanical architecture and hand coordination is challenging. It is not understood which biomechanical characteristics are responsible for hand coordination and what specific effect each biomechanical characteristic has. To explore this link, we first inspected the characteristics of hand coordination during daily tasks through a statistical analysis of the kinematic data, which were collected from thirty right-handed subjects during a multitude of grasping tasks. Then, the functional link between biomechanical architecture and hand coordination was drawn by establishing the clear corresponding causality between the tendinous connective characteristics of the human hand and the coordinated characteristics during daily grasping activities. The explicit functional link indicates that the biomechanical characteristic of tendinous connective architecture between muscles and articulations is the proper design by the Creator to perform a multitude of daily tasks in a comfortable way. The clear link between the structure and the function of the human hand also suggests that the design of a multifunctional robotic hand should be able to better imitate such basic architecture.

## Introduction

The human hand is an amazing instrument that can perform a multitude of functions, such as the power grasp and precision grasp of a vast array of objects. The excellent behaviors of the human hand are enabled by a highly complex structure, with 19 articulations, 31 muscles and more than 25 degrees of freedom (DOF) [1]. While the abundant functions are favorable, this complex structure also raises a challenging problem of how the human body controls such a large number of mechanical DOFs with ease and an absence of effort.

RETRACTED

Studies indicate that digits do not move alone in isolation of adjacent digits during functional activity [2], even when a specific movement requires an individual digit [3]. On the contrary, the movements of multiple digits are correlated, and movement information of the human hand is redundant, so that only a small number of components account for most variances [4]. The human hand adopts coordinated movements to reduce the number of independent DOFs and simplify the complexity of the control problem [5,6]. Thus, hand coordination affords humans the ability to flexibly and comfortably control the complex structure to perform numerous tasks. Hand coordination should indicate the mystery of the Creator’s invention.

There are two main factors that contribute to hand coordination: neurological functions and biomechanical constraints [7]. The neurological functions are controlled by the central nervous system (CNS) [8]. The CNS receives sensory information, such as smells, tastes, sounds, sights and tactile information, and responds to the information with an action, which can move different fingers simultaneously through the spillover of the neural drive to neighboring muscles [9]. Compared to the neurological functions, knowledge of the complex biomechanical architecture is more crucial to understanding hand coordination because mechanical functions can affect motor commands [10]. In the human hand, a single muscle does not always connect a single articular but rather has a unique connective architecture between muscles and articulations, such as the interconnection of a multi-tendon muscle with several articulations. Although many researchers have noted the effect of the biomechanical constraints on hand coordination [1,3,7,10], few have found a clear link between the biomechanical architecture and hand coordination. In this paper, we will explore such a functional link.

Before establishing the clear link between biomechanical architecture and hand coordination, we studied the characteristics of the coordinated movement of the human hand during grasping activities in daily living. As far as we know, considerable attentions have been devoted to investigating the characteristics of the coordinated relationships between fingers or joints using a multivariate statistical analysis of the kinematic data, which were collected from subjects during tasks or a period of natural movements [11–16]. However, in most of these studies the movement data are gathered from only a few grasping types while not covering various grasp tasks in daily life as much as possible. And the grasping tasks are also different in these research works. As discussed in this paper, the human hand adopts a distinctive coordinated control strategy for each task. It is apparent to get different coordinated relationships between joints from the movement data compiled by different tasks. Considering that the versatile ability to complete various tasks is a crucial advantage of the human hand, it is necessary to understand the basic characteristics of coordinated movement needed when various tasks are performed. Thus, we collected kinematic data from a sufficient number of tasks, which represented a variety of grasp tasks in daily life as much as possible, to explore the basic coordinated relationships between joints. In addition, cluster analysis was used to determine a network and detailed coordinated relationship among joints.

RETRACTED

After determining the basic characteristics of coordinated movement, we tried to find clear corresponding evidence of coordinated relationships from the biomechanical characteristics of muscular-articular connective architecture and to establish the functional link between the biomechanical architecture and the characteristics of hand coordination. Clear evidence would indicate that the muscular-articular connective architecture of the human hand is responsible for the basic dexterous control strategy for various tasks. This study explores a method to identify the proper explanation for the hand architecture of muscular-articular connections from the analysis of behavioral result.

## Materials and Methods

### Task paradigm

In daily use, grasping is the most common function of the human hand [7]. Many studies have focused on grasping to mimic the ability for artificial hands [17,18]. The human hand can grasp different objects of a vast range of sizes and shapes. People are more concerned with the tasks they wanted to accomplish than the sizes and shapes of objects in terms of the choice of grasp. This suggests that grasps could be categorized according to tasks instead of appearance [19]. An early attempt to characterize grasp was made by Napier [20]. He suggested that the diversity of grasp activities of the human hand could be composed of two basic functional modes: power grasp and precision grasp. The former is characterized by application of force with a large contact area between objects and the hand surface. In the latter, the objects are dexterously held with the tips of the fingers and thumb. Following Napier, many researchers have elaborated the two basic categories by proposing further subdivisions [19,21,22]. These subdivisions are based on the details of the tasks in terms of which group of fingers exerted force on the object and which part of the finger contacted the object [4]. Feix incorporated the grasp taxonomy from existing studies and developed a comprehensive taxonomy [23]. In particular, he considered the distinctiveness of the thumb and expanded the taxonomy to 33 different task types (as shown in S1 Fig). This finite taxonomy is able to allow a better description of the capabilities of the human hand. Therefore, the Feix taxonomy was chosen as our task paradigm.

RETRACTED

### Subjects

Thirty asymptomatic subjects (15 males and 15 females, 25 years old on average) participated in the experiment after providing written informed consent. None of the subjects had any known history of neurological or musculoskeletal problems that might affect their hand function. They also possessed no particular hand skill as a result of work or leisure activities, such as being proficient in playing the piano. Each subject was required to fill out a Edinburgh Inventory questionnaire to quantify their handedness on the laterality quotient scale [24]. A value of +100 indicated maximally right-handed, and a value of -100 indicated maximally left-handed. The laterality quotient for these subjects ranged from +68 to +100, and the subjects were all right-handed. The experimental protocol was approved by the ethics committee of the Tongji Medical College.

### Experimental procedure

Subjects were seated near the edge of a table and placed their right arm on the table in a comfortable posture. They were instructed to perform 33 types of tasks (S1 Fig) using a large number of objects, which were chosen from the most common objects in daily life and had a large range of sizes and shapes, such as cylinders, disks, spheres and cards. In each type of task, the subjects were asked to grasp three objects of different sizes or shapes separately, and each test was repeated on every object three times to depress random error. At the beginning of each trial, objects were placed beyond the subjects’ suitable reaching distance, and the subjects extended their right hand in a natural full extension. Upon hearing the “go” command (in Chinese), the subjects started to grasp the object at a self-paced speed. They were allowed to move the proximal arm in accordance with the hand motion during the experiment.

An instrumented glove (CyberGlove, Virtual Technologies, Palo Alto, CA, USA) with embedded resistive bend sensors was used to measure the joint angles of the hand during the grasping movement from the start command to the completion of the task. Before each subject was tested, the glove sensors were calibrated between sensor output and joint angle by establishing an approximate linear regression relationship [3,13]. Data from each glove sensor were sampled at 50 Hz and stored to a disk on a personal computer. As shown in Fig 1A, we recorded the data from 16 sensors, which consisted of the metacarpal-phalangeal (MCP), proximal inter-phalangeal (PIP) and distal inter-phalangeal (DIP) sensors for the four fingers (Index: I, Middle: M, Ring: R, Little: L) and the carpometacarpal (CMC), MCP, inter-phalangeal (IP) and abduction (ABD) sensors for the thumb (T). The MCP, PIP, and DIP sensors for the four fingers and the MCP and IP sensors for the thumb were applied to measure the flexion-extension (fe) movement (Fig 1B). It should be noticed that the CMC joint of the thumb is a compound joint and has two non-orthogonal rotation axes, which are located in different bones. The adduction-abduction (aa) axis passes through the proximal end of the metacarpal bone, while the fe axis intersects with the trapezium carpal bone [25]. The non-orthogonal and non-intersecting axes of the CMC joint made it difficult to measure the joint angles accurately using the instrument glove. An alternative method for the CyberGlove was to measure the angle of the thumb rotating across the palm and the angle between the thumb and index finger using CMC and ABD sensors to replace the two joint angles of the compound joint. Flexion and abduction were defined as positive, as shown by the rotating direction of the arrows in Fig 1B.

RETRACTED

**Fig 1:** CyberGlove sensor placement and corresponding kinematic model of human hand. (A) Placement of 16 sensors used in the CyberGlove (the image is adapted from Ingram 2008, with kind permission from Springer Science + Business Media). (B) Joints and the kinematic model of the human hand. Abbreviations: MCP, metacarpal-phalangeal; PIP, proximal inter-phalangeal; DIP, distal inter-phalangeal; CMC, carpometacarpal; IP, inter-phalangeal; ABD, abduction; T, thumb; I, Index; M, Middle; R, Ring; L, Little; fe, flexion-extension; aa, abduction-adduction.

### Data analysis

As mentioned previously, we used the CyberGlove to record the joint angles of the human hand from the 16 sensors, and each trial discretely sampled from the beginning time to the movement completion time during each task. A Butterworth filter was used to smooth the digitized sensor data and reduce the noise caused by the acquisition instrument. For each subject, data from all recording sessions of the *k*th task were concatenated to form a movement data $Q_{k}\in {ℜ}^{16\times n_{k}}$, where *n*_*k*_ represents the sample number of discrete joint angles during the respective task. All movement data **Q**_*k*_ of the 33 types of tasks for a subject were concatenated to create the movement dataset $Q\in {ℜ}^{16\times n}$ during the entire experiment.

RETRACTED

Principal components analysis (PCA) was employed to investigate the degree of the coordinated behavior among the joints of the human hand. This dimensional reduction method transformed the original dataset of correlated joint angle variables into a linear combination of new, uncorrelated variables called principal components (PCs). The PCs were derived as the eigenvectors of the covariance matrix computed from the joint angle dataset **Q**. Then, the PCs were ordered according to the percentage of variance explained by each component [26]. The first PC accounted for the greatest variation and gave the best fit to all of the movement data of the joint angles. The second maximized the variation excluding the first PC, and so on. The smaller numbers of PCs accounted for most variance, and a higher degree of coordinated movement existed among joints during the whole experiment of various tasks.

Correlation analysis was used to determine the coordinated relationships between joints. If two joints were coordinated, they would move synchronously with a certain relationship. The degree of the movement-coordinated relationship between joints could be described by Pearson’s correlation coefficient of the time-varying angular data. However, the absolute value of Pearson’s correlation coefficient was chosen as the measurement of the movement-coordinated relationship by ignoring the relative movement direction. We applied correlation analysis on different movement datasets composed of different tasks. At first, the movement dataset **Q**_*k*_ for each task was used to determine the coordinated relationships between joints. There were 16×(16–1)/2 = 120 variables of coordinated relationships between joints, and the average value of all variables was used to denote the general evaluation of the movement coordination. Next, the movement datasets for multiple tasks were pooled to analyze and obtain the common coordinated relationships for these tasks. To study the influence of richness of task type, different numbers of task types were chosen to comprise the pooled movement datasets and determine their respective common coordinated relationships. When choosing *m* number of tasks from the 33 tasks in S1 Fig, there were $C_{33}^{m}$ combination possibilities, and it was necessary to equalize all of the possibilities to give a statistical result. However, it was a time-consuming calculation to exhaust all possibilities because the number of possible combinations could reach 1.17×10^9^ when 16 types of tasks were chosen. Instead, we randomly selected 2000 types from all possible combinations except the conditions of choosing one or two types of tasks, which would have less than 2000 possibilities. Therefore, when choosing *m* number of tasks, the general evaluation of the coordinated relationship, called the mean movement coordination (MMC), was defined as

$$MMC=\left\{\begin{array}{c} \frac{1}{33}\sum_{c=1}^{33}(\frac{1}{120}\sum_{i,j}^{}\left|r_{ij}^{c}\right|)\;m=1\;\\ \frac{1}{528}\sum_{c=1}^{528}(\frac{1}{120}\sum_{i,j}^{}\left|r_{ij}^{c}\right|)\;m=2\;\\ \frac{1}{2000}\sum_{c=1}^{2000}(\frac{1}{120}\sum_{i,j}^{}\left|r_{ij}^{c}\right|)\;m>2\; \end{array}\right\},$$ (1)

where 1≤*i*<*j*≤16, $r_{ij}^{c}$ represents the correlation coefficient between the *i*th and *j*th joints in the *c*th possible combination under the condition of choosing *m* number of tasks as movement datasets.

RETRACTED

After comparing movement-coordinated relationships between tasks, we used correlation analysis on the movement dataset **Q** to explore the basic coordinated relationships between any two joints for various tasks. The agglomerative hierarchical clustering method was applied to obtain the detailed movement-coordinated relationships among the joints of the human hand. This clustering method started with the individual joint variables, and each joint variable acted as a separate cluster [27]. The absolute value of the correlation coefficient between every two joint variables, which described the movement-coordinated relationship, was taken as the similarity measurement between these clusters. The two most similar clusters were first merged to create a new cluster. In subsequent steps, the more similar clusters were continuously merged into a single cluster. The similarity between two clusters should be recalculated at each step, and the measure was defined as follows using the average linkage algorithm:

$$r_{UV}=\frac{\sum_{i\in U}\sum_{j\in V}\left|r_{ij}\right|}{N_{U}V_{V}},$$ (2)

where *r*_*ij*_ is the correlation coefficient between the i*th* element of cluster *U* and the j*th* element of cluster *V*. *N*_*U*_ and *N*_*V*_ represent the numbers of the elements in each cluster, respectively.

#### Statistical analyses

To provide a statistical description, we performed significance tests of our results in the correlation analysis and clustering analysis. In the correlation analysis, a one-tailed paired t-test was used to test whether the average value of the coordinated relationships in one task was significantly higher or lower than that in another task. The same test was employed in the case of comparing the coordinated relationships between different joint pairs. In the clustering analysis, the values of the movement-coordinated relationships across all subjects were averaged to conduct the cluster analysis by continuous agglomeration of similar clusters. In each agglomerative step, the similarity between clusters was the mean value of all subjects, and the two clusters with the highest value of similarity were grouped. The results appeared to indicate that the two clusters were more similar to one another than to other clusters. However, this result of clustering was based on the average value across subjects, and the two clusters in many subjects might be more similar to other clusters than to one another due to the individual differences. To test the statistical significance of such clustering results in every agglomerative step, we used a one-tailed paired t-test to separately test whether the similarity between the two agglomerative clusters was significantly higher than the similarity between the two clusters with each of the other clusters. The Bonferroni-Holm correction of the p value was used for multiple comparisons of the similarities [28], and the highest corrected p value was taken as the significance of each agglomerative result. The probability level of *p*<0.05 was chosen as statistical significance for each test.

RETRACTED

## Results

### Degree of coordinated movement among joints

The human hand is a complex and redundant system of coordinated movements that performs a variety of motions. Using the movement dataset of the human hand determined from the experimental paradigm (see Materials and Methods), the principal component analysis (PCA) obtained 16 principal components (PC) as the movement dataset, potentially spanning a 16-dimensional space. The percentage of variance accounted for the joint angles by each successive PC (bars in Fig 2) diminishes progressively, and the first few PCs can retain most of the movement information of the original joint variables. For example, the first three PCs account for 83.4±2.0% (mean ± standard deviations across subjects) of the variance, and the first seven PCs account for nearly 96.4±0.7% of the variance. This demonstrates that the movement datasets of joint angles are hyper-redundant. This result provides an insight into the highly coordinated movement among the joints in the human hand even when a lot of tasks need to be performed.

**Fig 2:** A Pareto chart for the variance explained by the movement dataset of joint angles. The bars illustrate the variance explained by each principal component (PC) from the PCA, and the line illustrates the cumulative variance explained by the retaining PCs. Error bars indicate standard deviations across subjects.

### Comparison of the coordinated movement between tasks

The human hand coordinates multiple joints to dexterously perform different tasks in different ways. The dexterous control strategy for each task can be described by the specific coordinated movement between joints, as shown in Fig 3. The values of 120 coordinated variables by pairwise combinations of 16 joints are distributed along the ring circle in each radar chart in Fig 3. The coordinated relationships concerned with the joints of thumb among the pairwise combinations of all 16 joints are shown in area 1, the coordinated relationships concerned with the joints of the index finger among the pairwise combinations of the remaining joints of the four fingers without the thumb are shown in area 2, and so on. The six tasks were chosen to represent the features of all tasks. The results in Fig 3 indicate that the human hand can apply different adjustments of coordinated relationships to realize a specific dexterous control strategy for different tasks, such as a local adjustment of the coordinated relationships concerned with the thumb joints (comparing Fig 3A and 3B), a wide range of adjustments of the coordinated relationships between joints (comparing Fig 3C and 3D), and adjustments based on the complexity of tasks (comparing Fig 3E and 3F with Fig 3A or 3B). An extended discussion about the comparison of coordinated relationships between tasks is presented in S1 Text. The adjustments make the movement-coordinated relationships between tasks have significant distinctions.

RETRACTED

**Fig 3:** Movement-coordinated relationships between joints of the human hand in each type of task. There are 16×(16–1)/2 = 120 variables of movement-coordinated relationships between every two of the 16 joints recorded in the movement dataset, and they are distributed along the ring circle in the radar chart. Area 1 represents the coordinated relationships regarding the joints of thumb and contains the internal relationships between the joints of the thumb and the external relationships between the joints of thumb and the other four fingers. Similarly, area 2 represents the coordinated relationships regarding o the joints of the index finger excluding the joints of the thumb, and so on. The coordinated relationships between all joints of the ring and little fingers are represented in area 4 of the chart. The amplitudes of the coordinated relationships are averaged across all subjects. The six tasks are chosen to represent the features of all tasks.

Not only for a single task, the joints of human hand are also coordinated during the movement of multiple tasks [14]. The coordinated relationships between joints for these tasks are called common coordinated relationships and can be derived from the pooled movement datasets composed of these tasks. The common coordinated relationships represent the dexterous control strategy for satisfying the functional requirements of these tasks. Although many investigators have studied common coordinated relationships between fingers or joints using kinematic data, which are collected from subjects executing some tasks or during a period of natural movements [11,13,16], most of these studies have been limited to a few types of different tasks. As discussed in the previous study, the human hand adopts a distinctive control strategy for each task, and it is apparent to get different common coordinated relationships between joints from the movement dataset composed of different tasks. When more tasks need to be performed, the common coordinated relationships for all of these tasks will change, but it is unknown whether the common coordinated relationships will always change with an increase in tasks. In other words, do constant and basic common coordinated relationships exist for the human hand when various tasks are performed? To answer this question, we studied the influence of richness of task type on the common coordinated relationships. When several tasks are chosen, the evaluation index of mean movement coordination (MMC, see Materials and Methods) is employed to show the general movement-coordinated relationships among joints. As shown in Fig 4, a significant trend is that the coordination drops with an increase in the number of task types despite the individual differences. When only one task is chosen, the value of the MMC is higher. However, the coordination drops rapidly when more tasks are added. This decrease of coordination indicates that the realization of more functions requires more independent movements. However, the coordination does not always decrease. The rate of decrease becomes quite slow and the MMC value turns into invariableness when many tasks are included, especially when more than 20 types of tasks are chosen, as shown in Fig 4. The invariable coordination shows that constant common coordinated relationships exist for human hand to perform various tasks. The characteristics of the invariable coordination also reflect the basic dexterous control strategy of the human hand to satisfy the functional requirement of various tasks.

RETRACTED

**Fig 4:** Relationship between the mean movement coordination (MMC) and the numbers of task types. It shows some representative results from several subjects. Abbreviate: SUBJ, Subject.

### Movement-coordinated relationships between joints during all the tasks

In the previous comparisons, each task had its own distinctive movement-coordinated relationships between joints to achieve their respective dexterous control strategies. When the movement datasets of 33 tasks were pooled to represent the movements of various tasks in daily life, their common coordinated relationships would remain invariable, and the common coordinated relationships revealed the inherent characteristics of the human hand. We analyzed the pooled movement dataset composed of these tasks to determine the detailed coordinated characteristic between joints to explore the basic dexterous control strategy of the human hand for various tasks.

The coordinated relationship for a joint pair was calculated by the correlation coefficient between the time-varying angular data. The values of movement-coordinated relationships for all combinations of the 16 joints were averaged across subjects and can be expressed by the matrix $R\in {ℜ}^{16\times 16}$. A graph (Fig 5) is used to represent the numerical value of the matrix by the grayscale in each square. The grayscale graph is then colored with pastel shades of pink to strength the visual effects, with pink representing higher coordination. The characteristics of coordinated relationships between each pair of joints in Fig 5 are discussed in the S2 Text.

**Fig 5:** Graphic description of coordinated relationships for joint pairs. The value of coordination was averaged across subjects and is denoted by the grayscale with pink in each square. The pink color indicates the higher coordination for the corresponding joint pair. The diagram is axisymmetric. Dashed and solid lines passing through squares are used to describe different areas for joint pairs. The joints and abbreviated names are shown in Fig 1.

An agglomerative hierarchical cluster analysis is used to explore the general movement-coordinated relationships among joints. The analysis from the averaged movement-coordinated relationships across subjects (the same values as in Fig 5) results in a tree structure (dendrogram) of relationships among all joint variables. The dendrogram (Fig 6) shows the continuously agglomerative process of the cluster method from the bottom up. The PIP joint of the ring finger and the PIP joint of the little finger first meet at a node among all joints. This denotes that the average coordination across subjects for these two joints is the highest among all the combinations of joint pairs. However, taking into account individual differences, the coordination for the PIP joint pair of the ring and little fingers is 0.9285 ± 0.0241 (mean ± standard deviations across subjects), and the coordination for the PIP joint pair of the middle and ring fingers is 0.9261 ± 0.0449. The coordination for the PIP joint pair of the ring and little fingers is not significantly higher than the coordination for the PIP joint pair of the middle and ring fingers (29, *t* = 0.25; *p* = 0.40). It suggests that the coordination for the PIP joint pair of the ring and little fingers may be lower than that between the middle and ring fingers in a considerable number of the subjects. Thus, the first clustering for the PIP joints of the ring and little fingers has no statistical significance. In the following clustering process, the PIP joints of the ring and little fingers meet the PIP joint of the middle finger at a higher height of node, and the three joints were clustered to a group. The coordination is 0.8753 ± 0.0511 between the old cluster of PIP joints of the little and ring fingers and the PIP joint of middle finger, which is also equivalent to the similarity measurement between clusters (*r*_UV_, see Materials and Methods). This coordination is significantly higher than the coordinated relationships between the old cluster with any others clusters in this agglomerative phase (corrected *p* = 0.013<0.05). The clustering of the three PIP joints has statistical significance, and all the significant clusters are marked under the respective clustering nodes in Fig 6.

RETRACTED

**Fig 6:** Dendrogram of the clustering of joints. This graphically shows the network of movement-coordinated relationships among the joints of the human hand. The lower branch nodes of the tree indicate better-coordinated relationships between the joints under the two branches. The significances of clustering are marked with * (p<0.05), ** (p<0.01) and *** (p<0.001) under the nodes.

Considering the significant clustering results from the top down in Fig 6, we can draw four main coordinated characteristics between joints during the movement of various tasks. First, an overall characteristic is that the joints of the four fingers are clustered into a group, while the joints of the thumb are clustered to one another. The coordinated relationship between the two groups is only 0.16 ± 0.05. The movements of the thumb joints have quite poor coordinated relationships with the joints of the four fingers. It should be noted that we ignored the result of a clustering group between the CMC and ABD joints of the thumb because they belong to a non-orthogonal and non-intersecting compound joint. Second, the joints of the four fingers are divided into two clusters, the PIP and DIP joints and the MCP joints. This demonstrates not only that the PIP and DIP joints in each finger are more coordinated than the MCP joint but also that all PIP and DIP joints of the four fingers are more coordinated than the MCP joints during the movement of various tasks. This coordinated characteristic indicates that the dexterous control of the human hand is not based on singer fingers but on joints. If control of the human hand was based on a single finger, the three joints of every finger should be more coordinated within one other than with the joints of the other fingers. The movement characteristic coincides with the functional need of the human hand to coordinate all joints to perform tasks in daily life more than to have selective control of the operation of individual fingers, such as for counting and playing the piano. Third, the movements of the joints of the index finger are distinct from the other joints of the middle, ring and little fingers. The joints of the index finger are separated from other fingers in both the cluster of the PIP and DIP joints and the cluster of the MCP joints of the four fingers (Fig 6). Fourth, the PIP joints of the middle, ring and little fingers are clustered in a group. The PIP joints are more coordinated among the PIP and DIP joints of the three fingers. In addition, to test whether these movement characteristics are related to the gender, we also group the movement data of female and male subjects to separately study their movement characteristics. As shown in S2 Fig, the significant clustering results in female and male subjects are the same as the results of the whole subjects (Fig 6), although there are some differences in the non-significant clustering nodes. The main movement characteristics are consistent between females and males.

RETRACTED

## Discussion

An important advantage that makes human hand superior to other animals is that the human hand can dexterously perform various tasks, and this unique ability can apparently facilitate the capacity for more effective tool making and tool use during the evolutionary process [29]. To explore the dexterous ability of the human hand, we adopted the reverse research method, going from the result to the reason. In previous work, we studied what basic movement characteristics are required for the human hand to perform multiple tasks dexterously. The following discussions are devoted to finding clear corresponding evidence to determine the reasons for hand coordination.

The movement characteristics of all joints of the human hand show that the joints of the thumb have lower coordinated relationships with the joints of the four fingers. The movement of the thumb is distinct from that of the four fingers. The flexor digitorum profundus (FDP) muscle is an important flexor muscle of the human hand and is located on the underside of the forearm (S3 and S4A Figs). In most non-hominoid primates, the FDP muscle separates five long tendons, and each attaches to one digit [30]. As shown in S4B Fig of a Barbary ape hand, the four fingers and thumb are interconnected by these long tendons of the FDP muscle. However, in the great apes (i.e., Pongo, Gorilla and Pan), the FDP tendon to the thumb is usually either vestigial or absent [31]. In humans, the FDP muscle only attaches to the four fingers, while the thumb has a separate long flexor muscle in the forearm called the flexor pollicis longus (FPL) muscle (S3 and S4A Figs). The presence of the FPL muscle is a specialization in humans and enormously increases the independence of the thumb. The movement characteristics of the human hand show that the thumb needs to be able to move independently of the other four fingers to perform various tasks. Fortunately, the presence of the FPL exactly satisfies the functional requirement and offers the human hand superior capacities to perform a variety of complex functions compared to other primates. In addition to the FDP muscle, the flexor digitorum superficialis (FDS) and extensor digitorum communis muscles are the other hand multi-tendon muscles. They only connect the four fingers as well, while the movements of the thumb joints are driven by exclusive muscles. The separate biomechanical structure of the thumb is reflected in the poor movement-coordinated relationships between the thumb and the four fingers.

RETRACTED

Another movement characteristic of the human hand is that the PIP and DIP joints of the four fingers are more coordinated than the MCP joins. The flexion motions of the DIP and PIP joints of each finger are primarily due to the separate actions of the FDP and FDS muscles [32]. The FDP muscle attaches to the distal phalanx of the finger with tendons (S5A Fig) and primarily generates motion at the DIP joint, while the FDS muscle inserts on the middle phalanx and primarily contributes to the flexion motion of the PIP joint [33]. However, flexion movement needs not only a synergist of flexor muscles but also an antagonist of extensor muscles to form an equilibration. An important extensor muscle is located in the forearm and performs via the long extensor tendon (S5A Fig). At the distal end of the metacarpal, the extensor tendon expands to form a hood (S5B Fig), which covers the MCP joint dorsally and warps around the sides of the metacarpal and proximal phalanx [34]. The extensor expansion soon splits into three bands, two lateral bands and a single central band, to attach to the distal and middle phalanges, respectively. Lateral bands collaterally pass on either side of the proximal phalanx and recombine again at the middle phalanx to attach to the distal phalanx. The central band passes down the middle of the finger along the back of the proximal phalanx and stretches to the base of the middle phalanx. The compound tendinous attachments of the extensor expansion connect the PIP and DIP joints and make the two joints rotate as a mechanism with one degree of freedom when the FDP is active, together with the taut central and lateral bands [35–37]. Detailed descriptions of the coupling principle can be found in the literature [35,38]. The specific structure of extensor expansion causes the movement of the PIP and DIP joints in each finger to be better coordinated. In addition, the flexion motions of the PIP and DIP joints for each finger are derived from the same muscles, FDP and FDS, which are two extrinsic flexor muscles (S3 Fig). About halfway down the forearm, both the FDP and FDS muscles narrow to form four separate tendons, which pass to their respective fingers. The same muscles connect the four fingers and carry out the coordinated movements of the DIP joints or PIP joints of the four fingers. In combination with the structure of extensor expansion, these anatomical structures lead to better-coordinated relationships among all PIP and DIP joints of the four fingers.

RETRACTED

The coordinated characteristics between the joints of the four fingers also suggest that the movements of the MCP joints have significant difference with the PIP and DIP joints. Flexion at the MCP joint is brought about primarily by the lumbrical muscles, aided by the tendons of the FDP and FDS as well as the interosseous muscles. Except for the same muscles for the PIP and DIP joints, such as the FDP and FDS muscles, the particular lumbrical muscles for the MCP joints increase the diversity of movement and result in the relative independence of the MCP joints compared to the PIP and DIP joints of the four fingers. Moreover, the intrinsic muscles of lumbrical and interossei have specific actions on the movement of the four fingers. These intrinsic muscles pass along the finger and insert into the extensor expansion near the MCP joint (S5 Fig). On the one hand, because of the tendon crossing the palmar side of the MCP joint, pulling of the interosseous and lumbrical muscles causes the flexion movement of the MCP joint. On the other hand, because these muscles join the extensor expansion, which crosses the dorsal side of the finger, pulling of the interosseous and lumbrical muscles also results in the extension movement of the PIP and DIP joints. The movement direction of the tendon is shown with the red arrows in S5A Fig. The structural features of these intrinsic muscles, which contribute to both flexion of the MCP joint and extension of the PIP and DIP joints at the same time, further increase the movement difference between the MCP joints and IP (PIP and DIP) joints during various tasks.

RETRACTED

The characteristics of coordinated movement between fingers indicate that the movements of the joints of index finger are distinct from the other fingers. Four fingers are connected by the FDP muscle. It ends in four tendons to flex the four fingers coordinately, but the part that acts on the index finger is usually distinct. The FDP has a muscle group common to the middle, ring and little fingers (S3 Fig) and the muscle bellies and tendons for these fingers are interconnected by areolar tissue and tendinous slips to some extent [39,40]. The tendon to the index finger often has its own belly and remains discernibly separate from the other fingers throughout its course from the muscle belly to the palm [41,42]. The conspicuous separation of the muscle belly and tendon for the index finger from the other fingers can be responsible for the specialization of the independent functions of the index finger, whereas the other three fingers work together.

The movement characteristics between the PIP and DIP joints of the middle, ring and little fingers show that the PIP joints of these fingers are more coordinated. When considering a single finger, the movement of the PIP and DIP joints is better coordinated during the performance of various tasks. The most intuitive solution to satisfy this characteristic is that the two joints are coupled by a mechanism and directly actuated by a muscle. In fact, each finger of the human hand has two different muscles to control the two joints separately. The better-coordinated relationship is guaranteed by the specific structure of the extensor expansion. The benefit of such a design is to give independent movement ability to the DIP joint apart from the simultaneous movement with the PIP joint. For example, the DIP joint can still move to adapt to an irregularly shaped object when the middle phalanx has contacted the object during a power grasp. The design of the driving mechanism provides the DIP joints of fingers with more independent movement to enhance the adapted ability of the human hand, while the PIP joints remain the better-coordinated relationships.

Therefore, all the characteristics of coordinated movement for various grasp tasks can be found the clear corresponding evidences from the muscular-articular connective architecture of the human hand. These characteristics of coordinated movement reflect the basic functional requirements for dexterous performance of various tasks. And the muscular-articular connective architecture of the human hand exactly meets such functional requirements. This suggests that there is no need for the human hand to control each joint independently. If there was not such biomechanical architecture, such as the separated connection of each articular from a single muscle, it would significantly increase the computational burden of the CNS to make up for the loss of the biomechanical architecture. Thus, the architecture is the biomechanical basis of the dexterous movement that provides the human hand with the amazing ability to perform a multitude of daily tasks in a comfortable way. In conclusion, our study can improve the understanding of the human hand and confirm that the mechanical architecture is the proper design by the Creator for dexterous performance of numerous functions following the evolutionary remodeling of the ancestral hand for millions of years. Moreover, functional explanations for the mechanical architecture of the muscular-articular connection of the human hand can also aid in developing multifunctional robotic hands by designing them with similar basic architecture.

RETRACTED

## Supporting Information

S1 Fig A hand wearing an instrumented glove demonstrates the 33 types of tasks in the Feix taxonomy. (TIF)

S2 Fig Dendrogram of the clustering of joints within the female (A) and male (B) populations seperately. This graphically shows the network of movement-coordinated relationships among the joints of the human hand. The lower branch nodes of the tree indicate better-coordinated relationships between the joints under the two branches. The significances of clustering are marked with * (p<0.05), ** (p<0.01) and *** (p<0.001) under the nodes. Despite there are some differences of the clustering nodes between female and male subjects, the significant clustering nodes are the same between them.
(TIF)

S3 Fig Flexor digitorum profundus and flexor pollicis longus muscles in the palmar view of forearm. The image is adapted from Gray, 1918.
(TIF)

S4 Fig Human and ape hands. (A) human hand. (B) barbary ape hand. This illustration of human hand can be regarded as the hand part in S3 Fig with covering the skin in the surface of digits. FDP muscle in the ape hand separates five long tendons and each attaches one digit. Compared to the ape hand, human hand has a particular FPL muscle to act the thumb. The image is adapted from the science photo library, with permission.
(TIF)

S5 Fig Anatomy of the finger of right hand. (A) Radial view of finger. (B) Dorsal view. Black arrows indicate pull of long extensor tendon; red arrows indicate pull of interosseous and lumbrical muscles; dots indicate axis of rotation of joints (the image is adapted from Netter Image, 2014, with permission).
(TIF)

S1 Text Comparison of the coordinated movement between tasks. (DOCX)

S2 Text Characteristics of coordinated relationships between joint pairs. (DOCX)

RETRACTED

## References

[1] van DuinenH, GandeviaSC. Constraints for control of the human hand. J Physiol. 2011;589(23):5583–93. doi: 10.1113/jphysiol.2011.2178102198620510.1113/jphysiol.2011.217810PMC3249034

[2] SoechtingJF, FlandersM. Flexibility and repeatability of finger movements during typing: analysis of multiple degrees of freedom. J Comput Neurosci. 1997;4(1):29–46. doi: 10.1023/A:1008812426305 904645010.1023/a:1008812426305

[3] Häger-RossC, SchieberMH. Quantifying the independence of human finger movements: comparisons of digits, hands, and movement frequencies. J Neurosci. 2000;20(22):8542–50. 1106996210.1523/JNEUROSCI.20-22-08542.2000PMC6773164

[4] SantelloM, FlandersM, SoechtingJF. Postural hand synergies for tool use. J Neurosci. 1998;18(23):10105–15. 982276410.1523/JNEUROSCI.18-23-10105.1998PMC6793309

[5] ChenWB, XiongCH, YueSG. Mechanical Implementation of Kinematic Synergy for Continual Grasping Generation of Anthropomorphic Hand. IEEE ASME Trans Mechatron. 2015;20(3):1249–63. doi: 10.1109/TMECH.2014.2329006

[6] LiK, NatarajR, MarquardtTL, LiZM. Directional Coordination of Thumb and Finger Forces during Precision Pinch. PLoS ONE. 2013;8(11):e79400 doi: 10.1371/journal.pone.0079400 2423612810.1371/journal.pone.0079400PMC3827381

[7] SchieberMH, SantelloM. Hand function: peripheral and central constraints on performance. J Appl Physiol. 2004;96(6):2293–300. doi: 10.1152/japplphysiol.01063.2003 1513301610.1152/japplphysiol.01063.2003

[8] InmanM. Making Hands Jive: How the Body Manages Hand Coordination. PLoS Biol. 2006;4(6):e196 doi: 10.1371/journal.pbio.0040196 2007659110.1371/journal.pbio.0040196PMC1457010

[9] CastielloU. The neuroscience of grasping. Nat Rev Neurosci. 2005;6(9):726–36. doi: 10.1038/nrn1744 1610051810.1038/nrn1744

[10] SantelloM, Baud-BovyG, JörntellH. Neural bases of hand synergies. Front Comput Neurosci. 2013;7 doi: 10.3389/fncom.2013.0002310.3389/fncom.2013.00023PMC361912423579545

[11] BraidoP, ZhangX. Quantitative analysis of finger motion coordination in hand manipulative and gestic acts. Hum Mov Sci. 2004;22(6):661–78. doi: 10.1016/j.humov.2003.10.001 1506304710.1016/j.humov.2003.10.001

[12] ChenWB, XiongCH, HuangXL, SunRL, XiongYL. Kinematic analysis and dexterity evaluation of upper extremity in activities of daily living. Gait Posture. 2010;32(4):475–81. doi: 10.1016/j.gaitpost.2010.07.005 2069216010.1016/j.gaitpost.2010.07.005

[13] IngramJN, KördingKP, HowardIS, WolpertDM. The statistics of natural hand movements. Exp Brain Res. 2008;188(2):223–36. doi: 10.1007/s00221-008-1355-3 1836960810.1007/s00221-008-1355-3PMC2636901

RETRACTED

[14] MasonCR, GomezJE, EbnerTJ. Hand synergies during reach-to-grasp. J Neurophysiol. 2001;86(6):2896–910. 1173154610.1152/jn.2001.86.6.2896

[15] d'AvellaA, PortoneA, FernandezL, LacquanitiF. Control of fast-reaching movements by muscle synergy combinations. J Neurosci. 2006;26(30):7791–810. 1687072510.1523/JNEUROSCI.0830-06.2006PMC6674215

[16] SantelloM, FlandersM, SoechtingJF. Patterns of hand motion during grasping and the influence of sensory guidance. J Neurosci. 2002;22(4):1426–35. 1185046910.1523/JNEUROSCI.22-04-01426.2002PMC6757566

[17] XiongCH, DingH, XiongYL. Fundamentals of Robotic Grasping and Fixturing: World Scientific; 2007.

[18] XiongCH, LiYF, DingH, XiongYL. On the dynamic stability of grasping. Int J Rob Res. 1999;18(9):951–8. doi: 10.1177/02783649922066682

[19] CutkoskyMR. On grasp choice, grasp models, and the design of hands for manufacturing tasks. IEEE Trans Rob Autom. 1989;5(3):269–79. doi: 10.1109/70.34763

[20] NapierJR. The prehensile movements of the human hand. J Bone Joint Surg. 1956;38(4):902–13.10.1302/0301-620X.38B4.90213376678

[21] KlatzkyRL, McCloskeyB, DohertyS, PellegrinoJ, SmithT. Knowledge about hand shaping and knowledge about objects. J Mot Behav. 1987;19(2):187–213. 1498805810.1080/00222895.1987.10735407

[22] EdwardsSJ, BucklandDJ, McCoy-PowlenJ. Developmental and Functional Hand Grasps: Slack Incorporated; 2002.

[23] FeixT, PawlikR, SchmiedmayerH-B, RomeroJ, KragicD, editors. A comprehensive grasp taxonomy Robotics, Science and Systems: Workshop on Understanding the Human Hand for Advancing Robotic Manipulation; 2009.

[24] OldfieldRC. The assessment and analysis of handedness: The Edinburgh inventory. Neuropsychologia. 1971;9(1):97–113. doi: 10.1016/0028-3932(71)90067-4 514649110.1016/0028-3932(71)90067-4

[25] ChangLY, MatsuokaY, editors. A kinematic thumb model for the ACT hand International Conference on Robotics and Automation; 2006 15–19 5 2006: IEEE.

[26] JolliffeI. Principal Component Analysis: Wiley Online Library; 2005.

[27] JohnsonRA, WichernDW. Applied multivariate statistical analysis. JohnsonRA, WichernDW, editors: Prentice-Hall, Inc.; 2007.

[28] HolmS. A simple sequentially rejective multiple test procedure. Scand Stat. 1979;6(2):65–70.

[29] MarzkeMW, MarzkeRF. Evolution of the human hand: approaches to acquiring, analysing and interpreting the anatomical evidence. J Anat. 2000;197(1):121–40. doi: 10.1046/j.1469-7580.2000.19710121.x1099927410.1046/j.1469-7580.2000.19710121.xPMC1468111

[30] DiogoR, RichmondBG, WoodB. Evolution and homologies of primate and modern human hand and forearm muscles, with notes on thumb movements and tool use. J Hum Evol. 2012;63(1):64–78. doi: 10.1016/j.jhevol.2012.04.001 2264095410.1016/j.jhevol.2012.04.001

RETRACTED

[31] DiogoR, WoodBA. Comparative Anatomy and Phylogeny of Primate Muscles and Human Evolution: CRC Press; 2012.

[32] PalastangaN, FieldD, SoamesR. Anatomy and Human Movement: Structure and Function: Elsevier Health Sciences; 2006.

[33] FokKS, ChouSM. Development of a finger biomechanical model and its considerations. J Biomech. 2010;43(4):701–13. doi: 10.1016/j.jbiomech.2009.10.020 1996214810.1016/j.jbiomech.2009.10.020

[34] Garcia-EliasM, AnK-N, BerglundL, LinscheidRL, CooneyWPIii, ChaoEYS. Extensor mechanism of the fingers. I. A quantitative geometric study. J Hand Surg. 1991;16(6):1130–6. doi: 10.1016/S0363-5023(10)80079-610.1016/s0363-5023(10)80079-61748761

[35] BuchnerHJ, HinesMJ, HemamiH. A dynamic model for finger interphalangeal coordination. J Biomech. 1988;21(6):459–68. doi: 10.1016/0021-9290(88)90238-2 320959110.1016/0021-9290(88)90238-2

[36] BrookN, MizrahiJ, ShohamM, DayanJ. A biomechanical model of index finger dynamics. Med Eng Phys. 1995;17(1):54–63. doi: 10.1016/1350-4533(95)90378-O 770434510.1016/1350-4533(95)90378-o

[37] LandsmeerJ. The coordination of finger-joint motions. J Bone Joint Surg. 1963;45(8):1654–62.14083140

[38] LeijnseJNAL, SpoorCW. Reverse engineering finger extensor apparatus morphology from measured coupled interphalangeal joint angle trajectories—a generic 2D kinematic model. J Biomech. 2012;45(3):569–78. doi: 10.1016/j.jbiomech.2011.11.002 2213418310.1016/j.jbiomech.2011.11.002

[39] StandringS, EllisH, HealyJ, JohnsonD, WilliamsA, CollinsP, et al Gray's Anatomy: The Anatomical Basis of Clinical Practice: Elsevier; 2005.

[40] DoyleJR, BotteMJ. Surgical Anatomy of the Hand and Upper Extremity: Lippincott Williams & Wilkins; 2003.

[41] KahleW, FrotscherM. Color Atlas of Human Anatomy: Thieme; 2003.

[42] GrayH. Anatomy of the Human Body: Lea & Febiger; 1918.

